# Comparison of Modified Broström Procedure with or without Suture Tape Augmentation Technique for the Chronic Lateral Ankle Instability

**DOI:** 10.1155/2022/6172280

**Published:** 2022-07-27

**Authors:** Ji Li, Wei Qi, Xing Yun, Yu Wei, Yang Liu, Min Wei

**Affiliations:** Senior Department of Orthopedics, The Fourth Medical Center of Chinese PLA General Hospital, No. 51, Fucheng Road, Haidian District, 100048 Beijing, China

## Abstract

**Purpose:**

To compare the clinical outcomes of the modified Broström repair (MBR) with or without suture tape augmentation (STA) for managing the chronic lateral ankle instability.

**Methods:**

72 patients with chronic lateral ankle instability treated at our hospital from January 2018 to July 2019 were included, with 37 patients receiving the MBR and 35 treated by the MBR with STA. The clinical efficacy of the two techniques was assessed in terms of VAS, AOFAS, and Karlsson scores and by physical examination in follow-ups.

**Results:**

In all 72 patients, operations were successful, and the patients were followed up for 29.3 months on average (range, 24-43 months). There were no significant differences in preoperative pain, AOFAS, and Karlsson scores between the two groups. Compared with preoperative findings, all the functional scores were significantly improved in both groups 3 months after the operation and at the last follow-up. Three months after the operation, the STA group had significantly lower VAS and higher AOFAS scores than the isolated MBR group, suggesting that patients in the STA group suffered less pain and achieved better functional improvement. However, the VAS and functional scores at the last follow-up and the Karlsson score at 3 months postoperatively showed no intragroup difference in both groups.

**Conclusion:**

MBR with or without STA could achieve good results for the treatment of chronic lateral ankle instability. Compared with the widely used MBR, combining with STA may be more effective in promoting rehabilitation in early term.

## 1. Introduction

Currently, the sports-related injuries have been steadily on the rise. Among the injuries, lateral ankle sprains remain the most common one in most sporting activities [1]. Up to 10-20% of patients with acute ankle sprain later develop chronic ankle instability [2, 3]. Without timely and effective treatment, ankle instability not only significantly affects the patient's exercise ability but also leads to secondary diseases such as arthritis.

The modified Broström technique has already been accepted as the preferred procedure for the treatment of chronic ankle instability [4, 5]. Multiple studies reported that satisfactory clinical outcomes were accomplished after the Broström surgeries [6, 7]. Patients, especially those with high demands on exercise, wish to return to activity as soon as possible. Nonetheless, the ankle after Broström surgery needs to be immobilized for 4-6 weeks before rehabilitation starts since the efficacy relies on maturation of the native tissues [8, 9]. The tissues may take four to six months to recover before an athlete can return to activity with a low risk of reinjury [10, 11]. Besides, recently, some researchers doubt that the ankle joint stability can last long after the Broström operation [12, 13]. In recent years, some other techniques have been introduced for the treatment of chronic ankle instability. One procedure is the ligament augmentation using suture tape as internal brace to reinforce the attenuated ligaments [4]. While several biomechanical studies reported the mechanical superiority of the augmented anterior talofibular ligament reconstruction using suture tape over other alternatives [14, 15], this technique has not been widely used in clinical practice.

In the present study, the modified Broström procedure with or without the ligament augmentation technique using suture tape was used to treat the chronic ankle instability, and comparison was made between the two techniques in terms of the clinical outcomes, with an attempt to determine whether the suture tape technique could accelerate rehabilitation while, at the same time, protect the repaired ligament in short-term. We hypothesized that both techniques could attain good clinical outcomes, and the augmentation with a suture tape would allow accelerated rehabilitation in early term postoperatively.

## 2. Materials and Methods

The approval for the clinical trial was obtained from the ethics committee of our institution. The inclusion criterion was patients with chronic lateral ankle instability for more than 6 months. Patients were excluded if they had a BMI over 30, abnormal cavovarus foot alignment, concomitant ankle pathologies requiring additional surgeries, neuromuscular disorders, generalized ligamentous laxity (Beighton score > 4), and previously received ankle surgeries. Physical examination and MRI were performed to evaluate the stability and injuries of ankle.

This study examined the records of 117 patients with ankle instability, including 93 patients receiving surgeries from January 2018 to July 2019 in our hospital, which were all performed by a senior surgeon (WM). Among the surgically treated patients, 21 patients (including 12 with injury of tibiofibular syndesmosis or other concomitant ankle pathologies requiring additional surgeries, 2 with BMI over 30, and 7 with generalized ligamentous laxity) were excluded against the exclusion criterion. Eventually, 72 patients were included, and the 37 cases that received treatment with the modified Broström repair procedure were designated the MBR group. The other 35 cases surgically were treated with modified Broström repair procedure and suture tape augmentation, who are assigned to an STA group. All patients were preoperatively confirmed to have lateral ankle ligament injuries by means of MRI. All patients with conspicuous ankle instability were confirmed by the manual varus and anterior drawer stress test in comparison to the contralateral ankle.

### 2.1. Surgical Technique

The patient was placed in the lateral decubitus position and subjected to general anesthesia. Anteromedial, anterolateral, and accessory anterolateral portals were created for a diagnostic arthroscopy. Thorough inspection was performed for concomitant injuries. A motorized shaver and a radiofrequency blade were used to remove hyperplastic synovial membrane, damaged cartilage, and the loose body, among others. After creation of working space, the isometric point for anterior talofibular ligament (ATFL) in distal fibula and talar neck was cleaned, and cortical abrasion was applied. In the current study, 31 patients (17 in ST group and 14 in MB group) received arthroscopic synovectomy for soft tissue impingement syndrome, 9 patients (5 in ST group and 4 in MB group) underwent arthroscopic debridement for mild chondral lesions, and in 2 patients (2 in MB group), the loose bodies were taken out.

In the MBR group, after identification of remnants of lateral ligament complexes distal fibula was prepared, a cortical abrasion was applied, and two 2.3 mm PEEK suture anchors (Smith & Nephew) were inserted at footprints of the ATFL in the lateral malleolus. Lateral ligaments and articular capsule were reattached with suture anchors, and then the residual tissue in the proximal part including fibular periosteum was imbricated to the articular capsule.

In the STA group, two incisions were made at the anteroinferior border of the lateral malleolus and the lateral surface of the talar neck, respectively. A drill hole was made at the footprint of the ATFL on the talus, and the 3.5 mm SwiveLock anchor with FiberTape (Arthrex, Florida, America) was inserted. The second SwiveLock anchor and two 2.3 mm PEEK suture anchors were inserted into the footprint of the ATFL on the fibula, and the suture tape with maximal tension was securely fixed by a SwiveLock anchor. Then, the modified Broström repair was performed. Special attention was paid to insertion depth and direction to avoid penetration into the articular surface or retromalleolar groove. The remnants of FiberWire suture tape were cut out, level with the knotless suture anchors. The skin was then closed.

### 2.2. Postoperative Protocols

The two groups were on the same rehabilitation protocol. For 2 weeks after operation, a short leg cast was applied, and the patient was allowed to ambulate without weight bearing. In 3-4 weeks, the passive range of motion (ROM) training and partial-weight bearing ambulation should be conducted. From weeks 4 to 12, the cast was removed, and active ROM exercises, proprioception training, and gradually increasing weight bearing to full-weight bearing ambulation were permitted with an ankle brace worn for protection.

### 2.3. Clinical Evaluation and Follow-Up

Patients were followed up in our outpatient department 1, 3, 6, 12 months after surgery, and every 6 months thereafter. At every follow-up, to better evaluate the ankle stability and the recovery of ankle function, ROM, physical examinations (e.g., anterior drawer test) were performed in every follow-up. Scoring systems were used at 3 months and after follow-ups. Validated scoring systems for measuring chronic ankle instability were used, including VAS, AOFAS, and Karlsson scoring scale. Radiographs were taken immediately after surgery and at every follow-up to assess the ankle stability and the status of anchors. All preoperative and postoperative radiographic evaluations and all clinical assessments were conducted by observers who were not involved in patient care. Observers in this study were doctors working in our department and have in-depth knowledge of the disease, the surgery, and the scoring systems.

## 3. Results

Patients were followed up for 29.3 months on average (range, 24–43 months). Complete follow-up was achieved for all patients in both groups. These patients received complete serial physical and radiological examinations (Figure 1) and functional evaluations. Both groups were well matched with regard to the basic data (Table 1). Postoperative follow-up results of the two groups were comparable (*P* > 0.05). The preoperative manual varus and anterior drawer stress test, performed under anesthesia, were positive in all patients. Operations were successful in all 72 patients. The patients did not develop serious intraoperative complications or early postoperative complications, such as infection, thrombosis, joint fibrosis or adhesions, or implant failure.

Table 2 shows that there were no significant differences in preoperative pain, AOFAS, and Karlsson scores between the two groups. Compared with preoperative findings, all of the functional scores were significantly improved in both groups at 3 months postoperatively and at the last follow-up. Compared with the findings 3 months after operation, all of the functional scores were significantly improved in both groups at the last follow-up. At 3 months postoperatively, VAS was significantly lower, and the AOFAS score was significantly higher in the SAT group than that in the MBR group, indicating that patients in the STA group experienced less pain and had better function. However, the VAS and functional scores at the last follow-up, and the Karlsson score at 3 months after operation exhibited no intragroup difference between groups.

## 4. Discussions

Different techniques have been employed for the treatment of chronic lateral ankle instability. The modified Broström repair has been the most common and the gold-standard primary surgical technique for the lateral ankle ligament complex [5, 16]. In this study, the group of patients who underwent Broström repair showed significantly better clinical outcomes in terms of the pain, AOFAS, and Karlsson scores compared preoperatively. The results of the present work were similar with previous findings [17]. Nevertheless, in recent years, several follow-up studies reported that the Broström repair might fail to offer protection in the long term. Waldrop et al. suggested that the repaired lateral ligament after Broström technique was weaker than the natural, uninjured ligament, with only about 50% of the strength being restored by the procedure [18]. Kirk and colleagues reported that unprotected movement after the Broström repair could lead to a significant protracted rehabilitation and failure of the operation [19]. It may not be safe enough for the patients receiving Broström repair to undergo rehabilitation program in early postoperative period. In the recent years, the durability of the Broström repair technique for the treatment of lateral ankle stability has aroused some concerns. Xu and Lee reported that patients with ligamentous laxity had unsatisfactory outcomes in the long-term follow-up [12]. Maffulli et al. showed that 26% of patients abandoned all athletic activities, and 16% decreased their activity level after the Broström repair surgery [13]. Therefore, the Broström repair may not suffice to offer adequate improvement for patients who want to return to sports activities early and have a high exercise requirement, and other surgical alternatives with higher fixing strength are needed.

The ligament augmentation using suture tape as an internal brace to reinforce the attenuated ligaments was recently introduced for the treatment of chronic ankle instability. In theory, the STA technique may attain better stability due to the existence of suture tape than the traditional Broström repair. Although there was no direct ligament repair in isolated STA procedure, the restoration of ankle stability might contribute to the healing of attenuated ligaments. Several biomechanical studies reported the use of suture tape to reconstruct the anterior talofibular ligament had mechanical advantages over other procedures [14, 20]. Cho et al. reported excellent results in 28 patients with systemic generalization using InternalBrace™ augmentation for a Broström repair, and patients showed no signs of laxity over time [21]. Viens et al. also conducted a biomechanical study and found that use of InternalBrace™ to enhance Broström repair [22] yielded satisfactory results. In the present work, the patients undergoing STA showed significantly better clinical outcomes in terms of the pain relief, AOFAS, and Karlsson scores and the results of postoperative anterior drawer test, as compared with preoperative findings. In comparison with the traditional MBR technique, the STA method showed equally satisfactory outcomes at the last follow-up, and the finding was similar with the results of previous studies. Cho et al. reported that lateral ankle ligament augmentation using suture tape could accomplish clinical outcomes similar with the modified Broström repair for young female patients [23]. Ulku et al. found that, in an intermediate-term follow-up, arthroscopic lateral ligament augmentation with suture tape showed clinical outcomes comparable to arthroscopic Broström repair for the treatment of chronic ankle instability [24]. Additionally, the use of suture tape did not significantly increase the operative time. However, in the present work, at 3 months after operation, the STA group registered lower VAS scores but higher AOFAS scores, and most patients reported feeling stable and return to sports activities earlier. In our follow-up study, we even found that several patients felt sufficient stability and wanted to return to sports one month after operation. We believed that STA might be more effective in promoting rehabilitation at an early term.

However, complications after ligament reconstruction with synthetic materials cannot be ignored, such as immune response, synovitis caused by fragment dispersion, and recurrent instability due to mechanical failure. One case of chronic inflammation induced by foreign body reaction was reported in the aspect of suture enhancement of unstable ankle joint [25]. In this study, the follow-up max to 43 months revealed no suture tape-related immune complications.

### 4.1. Limitations

This study had several limitations. First, this was a nonrandomized retrospective study, the follow-up time was relatively short, and the sample size was small, which might increase the risk of type II error. A randomized controlled trial with a larger sample size and longer follow-up period is warranted in future. Second, the quality of physical examinations might vary with different examiners, and the results might be inaccurate. Moreover, no inter- or intraobserver reliability/variability was reported in this study. Third, stress radiographs and measurement of talar tilt angle can better reflect the lateral stability of ankle, but they were not taken in the study. Fourth, we used the same postoperative rehabilitation protocol for the two groups in this study, and different rehabilitation programs might be necessary in the future due to differences in the early stability.

## 5. Conclusion

Both MBR and STA could achieve good results in the treatment of chronic lateral ankle instability. Compared with the widely used MBR technique, the STA might be more effective in promoting rehabilitation at an early term.

## Figures and Tables

**Figure 1:** Preoperative and postoperative imaging of patients: (a, b) the preoperative radiography and MRI of patient in MBR group, respectively; (c, d) the postoperative radiography and MRI of the same patient in MBR group, respectively; (e, f) the preoperative radiography and MRI of patient in STA group, respectively; (g, h) the postoperative imaging of the same patient in STA group, respectively. The white arrows in (b) and (f) are the injured ligament, and the white arrows in (d) and (h) are the repaired ligament.

**Table 1:** Comparison of patients' data of the two groups.

Item	Group		Statistic	*P* value
	MBR (*n* = 37)	STA (*n* = 35)		
Gender (male/female)	21/16	19/16	*ꭓ* ^2^ = 0.182	NS (0.675)
Age	28.3 ± 5.7	31.2 ± 6.3	*t* = −0.937	NS (0.332)
Injury mechanism (sport/fall/traffic accident)	26/3/8	21/4/10	*ꭓ* ^2^ = 0.457	NS (0.829)
Affected limb (left/right)	13/24	10/25	*ꭓ* ^2^ = 0.118	NS (0.731)
Follow-up period (months)	30.6 ± 9.4	27.5 ± 10.7	*t* = −0.834	NS (0.816)
Operative time	71.3 ± 14.5	79.2 ± 18.1	*t* = −0.983	NS (0.149)

Data are presented as n or 95% confidence intervals. *t* and *ꭓ*^2^ are the corresponding statistics in independent-sample *t*-test and *ꭓ*^2^ test, respectively. NS: no significant difference.

**Table 2:** Comparison of functional scores between the 2 groups.

Item	Group		*t* value	*P* value
	MBR	STA		
VAS				
Preoperative	5.17 ± 1.36	5.34 ± 2.42	0.564	NS (0.575)
3 months	3.35 ± 1.56*a*	2.71 ± 0.98 *a*	2.067	0.042
The last follow-up	1.70 ± 0.99 *a*, *b*	1.57 ± 1.31 *a*	0.480	NS (0.633)
	*F* = 73.747, *P* < 0.001	*F* = 58.7, *P* < 0.001		
AOFAS				
Preoperative	54.03 ± 6.63	51.06 ± 8.33	1.679	NS (0.098)
3 months	72.11 ± 12.53 *a*	79.63 ± 15.77 *a*	-2.247	0.028
The last follow-up	86.62 ± 15.24 *a*, *b*	87.63 ± 15.16 *a*, *b*	-0.821	NS (0.415)
	*F* = 29.613, *P* < 0.001	*F* = 43.1, *P* < 0.001		
Karlsson score				
Preoperative	44.92 ± 9.22	41.54 ± 10.44	1.535	NS (0.129)
3 months	59.24 ± 8.82 *a*	62.11 ± 7.22*a*	-1.506	NS (0.137)
The last follow-up	73.27 ± 11.38 *a*, *b*	75.07 ± 8.11 *a*, *b*	-0.908	NS (0.481)
	*F* = 59.60, *P* < 0.001	*F* = 52.3, *P* < 0.001		

^a^There is significant difference compared with preoperatively. ^b^There is significant difference compared with 3 months postoperatively.

## Data Availability

The dataset supporting the conclusions of this article is included within the article. All data are fully available from the corresponding author on reasonable request.
